# Self-Attention-Guided Recurrent Neural Network and Motion Perception for Intelligent Prediction of Chronic Diseases

**DOI:** 10.1155/2021/6382619

**Published:** 2021-10-27

**Authors:** Baojuan Ma, Fengyan Zhang, Baoling Ma

**Affiliations:** ^1^Physical Education Department, Shijiazhuang Information Engineering Vocational College, Shijiazhuang 05000, Hebei, China; ^2^Physical Education and Health College, Hebei Normal University of Science and Technology, Qinhuangdao 066004, Hebei, China

## Abstract

Parkinson's disease is a common chronic disease that affects a large number of people. In the real world, however, Parkinson's disease can result in a loss of physical performance, which is classified as a movement disorder by clinicians. Parkinson's disease is currently diagnosed primarily through clinical symptoms, which are highly dependent on clinician experience. As a result, there is a need for effective early detection methods. Traditional machine learning algorithms filter out many inherently relevant features in the process of dimensionality reduction and feature classification, lowering the classification model's performance. To solve this problem and ensure high correlation between features while reducing dimensionality to achieve the goal of improving classification performance, this paper proposes a recurrent neural network classification model based on self attention and motion perception. Using a combination of self-attention mechanism and recurrent neural network, as well as wearable inertial sensors, the model classifies and trains the five brain area features extracted from MRI and DTI images (cerebral gray matter, white matter, cerebrospinal fluid density, and so on). Clinical and exercise data can be combined to produce characteristic parameters that can be used to describe movement sluggishness. The experimental results show that the model proposed in this paper improves the recognition performance of Parkinson's disease, which is better than the compared methods by 2.45% to 12.07%.

## 1. Introduction

Parkinson's disease (PD) [1, 2] is the second most common chronic central nervous system disease in the elderly population [3–5]. The loss of neuronal function is the most noticeable feature, and it has a significant impact on a person's motor function. In practice, this symptom affects a higher percentage of the elderly, and those over the age of 60 are more susceptible to the disease, with the proportion of patients under the age of 40 being relatively low. The treatment cycle of this disease is very long, and there is still a lack of very effective treatment methods [6]. Therefore, it will bring serious negative effects to the patient's family harmony and the stable operation of the society. Therefore, in order to better solve this problem, the initial auxiliary diagnosis [7, 8] of patients has very important practical significance.

There is currently no reliable method for detecting early-stage Parkinson's disease [9]. Most patients do not seek medical help in a timely manner and are unaware of the disease's existence due to a lack of comprehensive knowledge about Parkinson's disease. The symptoms of Parkinson's disease are frequently misdiagnosed as signs of aging. Parkinson's disease has a 60 percent delayed treatment rate due to a lack of early intervention and treatment [10]. Parkinson's disease is currently diagnosed primarily through clinical symptoms, which are highly dependent on clinician experience. As a result, there is a need for effective early detection methods.

Neuroimaging technology [11–14] is frequently used to quantify the loss of neurons in different areas of the brain to achieve the goal of detecting PD in order to better diagnose early PD. Magnetic resonance imaging (MRI) [15–18], functional magnetic resonance imaging (fMRI), and positron emission computed tomography (PET) [19] are some of the most commonly used neuroimaging technologies. PET has the disadvantages of low spatial resolution and high cost, while the other two imaging technologies are radioactive while in use. As a result, doctors will need a noninvasive, high-resolution method to track the progression, progression, and treatment of neurodegenerative diseases. According to current research, MRI has the advantages of high spatial resolution, noninvasiveness, low cost, and wide availability and can be used for the diagnosis of PD.

The application of artificial intelligence [20–22] in many fields has been confirmed with the development of machine learning [23–25]. More research [26–28] is currently focusing on proposing advanced machine learning technologies to solve practical applications [29]. Artificial intelligence also has a large market and potential in the medical field. Medical image recognition, for example, can assist doctors in reading patient images more quickly and accurately. Medical services such as clinical diagnosis assistant systems, for example, are used in early screening and diagnosis, rehabilitation, and surgery risk assessment scenarios, among other things. Therefore, the use of MRI images and machine learning algorithms to detect early PD is very promising. Recently, domestic and foreign scholars have proposed a method of combining brain images and machine learning to achieve the purpose of automatically predicting and evaluating the pathological stage, and there are many studies on PD. However, most of these algorithms only classify PD and normal control group. There are not many auxiliary diagnosis algorithms for early PD, and the accuracy of the classification algorithm for early PD and normal control group has room for improvement at this stage. Therefore, the research of efficient and accurate PD early feature selection and classification algorithms is of great significance to realize the early diagnosis of PD.

Furthermore, a common Parkinson's disease dyskinesia symptom is bradykinesia, and it is important symptom for determining the disease's diagnosis. Bradykinesia is a symptom of Parkinson's disease that affects nearly all patients and interferes with their daily activities, and it is drug-sensitive. The most common clinical manifestations are slow movement, difficulty moving, and loss of active movement ability. Motor retardation in the upper limbs can make it difficult to control fine daily activities such as typing, writing, and buttoning buttons with the hands. In the lower extremities, slow motion usually causes the foot to drag on the ground. In severe cases, it can lead to a panic and freezing gait (freezing is manifested as a sudden and short-term inability to move). The freezing gait is the most common cause of falls and increases significantly. It increases the risk of hip fracture. Other symptoms of motor retardation include decreased spontaneous movement, dysphagia, salivation, speech disorders, decreased facial expressions, decreased blinking, and decreased arm swing when walking. The evaluation of bradykinesia usually involves the patient performing repetitive, rapid, and alternating movements. Commonly used movements include finger tapping, hand clenching, hand pronation-supination, and heel up. This article is based on the wearable inertial measurement unit to carry out an objective quantitative assessment of the symptoms of bradykinesia, which can assist doctors in diagnosing Parkinson's disease and help reduce the medical costs of patients, thereby reducing the burden on patients and their families.

The main contributions of this article are as follows:

1. This paper proposes a novel intelligent predictive analysis model for chronic diseases based on self-attention-guided recurrent neural networks and motion perception, which is crucial for achieving early diagnosis of Parkinson's disease.
2. To classify and train the five brain region features extracted from MRI and DTI images, the proposed model employs a combination of self-attention mechanisms and recurrent neural networks. At the same time, it collects clinical data and motion data using wearable inertial sensors that can be worn on the body. The data are used to extract the characteristic parameters that can be used to characterize slow motion.

The following is how the rest of the paper is organized.  Section 2 examines some related work. In Section 3, some details about the proposed algorithm's principles and related submodules are presented. The experimental results are detailed in Section 4. In Section 5, the study's conclusion is presented.

## 2. Background

With the increasing incidence of Parkinson's disease, the problem of early PD detection has gradually become a new research hotspot that has attracted much attention in recent years. It belongs to the category of human activity recognition and is closely related to disciplines such as engineering, sports mechanics, and neuroscience. Some scholars have carried out a series of work on the extraction of physiological characteristics, motion characteristics, and the design of detection algorithms. In terms of feature extraction, the motion characteristics of PD patients have the following characteristics: (1) the stride length gradually decreases; (2) the joint range of the hip, knee, and ankle joints is greatly reduced; (3) the disordered time of the gait cycle control; (4) high-frequency alternating trembling leg movements.

Although there have been some studies using motion sensors to detect PD, the research work of many scholars is mainly focused on feature extraction and algorithm design. There are few studies on how to achieve the most effective system design, that is, to select the optimal sensor type, number, and deployment location. Considering the cost of deployment, a trade-off must be made between installing the least number of sensors and collecting the most information. Most studies use a single three-axis accelerometer, or combine it with a gyroscope, or combine it with a magnetometer to detect PD. Regarding the position where the patient wears the sensor, most studies use only one position. The tibia and waist are the most common placement locations for sensors. The rest include feet, knees, thighs, wrists, forearms, pants pockets, belly button, chest, and scalp. In addition, although many scholars have used machine learning algorithms to automatically identify PD, they have not discussed some important parameters that affect model performance and efficiency, such as the ratio of frozen gait to normal gait sample size in the training set and the size of the time window. Since frozen gait is difficult to collect sample size compared to normal gait, how to balance the ratio of the two to obtain the best classifier becomes a research focus of this article.

In addition, in the clinical setting, MRI diagnoses PD by evaluating structural and functional abnormalities. In order to achieve high-precision diagnosis, people try to design a computer-aided decision support system to realize automatic analysis of medical images. Extracting clinically relevant features from these images and helping to distinguish different disease categories is the key to achieving high classification accuracy. With the development of machine learning and data-driven analysis, the application of artificial intelligence in many fields has been affirmed. In the medical field, artificial intelligence also has huge potential and market. For example, medical image recognition helps doctors read patient images faster and more accurately and is effectively used in early screening, diagnosis, and surgical risk assessment. Recently, scholars at home and abroad have proposed a large number of studies using brain images and machine learning to automatically predict and evaluate pathological stages.

Recognizing healthy people or PD patients from subject images is a binary classification problem, which is very suitable for the implementation of machine learning (ML) technology. Medical data sets contain incomplete, inaccurate, and sparse information, so for the classification of these data, machine learning plays a vital role. With the rise of big data and artificial intelligence, neuroimaging classification methods increasingly use machine learning-related algorithms. These technologies can automatically extract a lot of information from the image set without preassuming the location of the information in the image. Many studies have evaluated the diagnostic value of these technologies, such as the diagnosis of Alzheimer's disease and mild cognitive impairment and have shown good research results. There is currently a study using supervised machine learning to perform individual differential diagnosis of PD and PSP on MRI, which is based on the combination of PCA and SVM with feature extraction technology. The current machine learning algorithms used for PD diagnosis mainly include principal component analysis, linear discriminant analysis, and nonnegative matrix factorization. Usually, these features are input into algorithms based on supervised learning, such as support vector machines (SVM) for feature classification.

## 3. Methodology

### 3.1. Feature Extraction

Generally speaking, brain image data have the characteristics of high dimension and relatively limited sample, which leads to the decline of the performance of decision model. Therefore, dimensionality reduction is needed for feature data. Dimension reduction is a preprocessing method for high-dimensional feature data, which preserves some important features of high-dimensional data and removes noise and unimportant features, so as to achieve the purpose of enhancing data processing efficiency. PCA and LDA are the most commonly used dimensionality reduction methods in Parkinson's disease classification algorithms. The feature of PCA is that the extracted features can accurately represent the sample information, so that the loss of information is very small. The feature of LDA is the feature after feature extraction. The accuracy of classification results should be high, which cannot be lower than that of the original feature classification. According to the characteristics of brain images, this study only needs to extract the best feature matrix with high correlation to reduce the dimension, so the PCA feature extraction method is adopted in this study.

### 3.2. Motion Data Collection Based on Inertial Sensors

To obtain effective PD personnel slow motion sample data, it is necessary to design a detailed and complete experimental data collection plan prior to data collection in order to ensure the smooth progress of the experiment. The experiment plan includes the experimental task design, experimental site design, experimental collection equipment and wearing parts, and object screening, as well as sample object design and data collection.

#### 3.2.1. Design of the Acquisition System

Fingers, wrists, waist, thighs, and ankles are the most common motion signals captured by the slow motion signal acquisition system. The signal collection system consists of a collection module with inertial sensors integrated. Velcro straps secure all collection modules to both hands' index and thumb fingers, wrists, thighs, ankles, and waist. The inertial sensors are worn in the positions as shown in Figure 1.

#### 3.2.2. Wearable Device Design

The acquisition module is mainly used to acquire the three-dimensional motion information of the human body. This research selects two inertial sensors as the acquisition module according to the different wearing positions. The sampling frequency of all the acquisition modules is 100 Hz.

The LPMS-B2 sensor from Japan's LP-RESEARCH company is used in the body node. A three-axis acceleration sensor, a three-axis gyroscope, and a three-axis magnetometer are all integrated into the sensor, allowing it to calculate the sensor's attitude direction and linear acceleration in real time. The low-power Bluetooth 4.1 (BLE) wireless transmission is used, and the on-board memory is 32M. The measured motion signal can be recorded in real time.

### 3.3. Recurrent Neural Network

Recurrent neural network (RNN) refers to a structure that recurs over time. It is widely used in many fields such as natural language processing and speech and image. The biggest difference between the RNN network and other networks is that RNN can achieve a certain “memory function” and is the best choice for time series analysis, just as human beings can better understand the world with their own past memories. RNN also implements this mechanism similar to the human brain, which retains a certain amount of memory for processed information, unlike other types of neural networks that cannot retain memory for processed information.

We can see the parameters in the RNN network from Figure 2. Here, only the behavior and mathematical derivation of the network at time *t* are analyzed. At time *t*, the network ushered in an input *x*_*t*_ and the neuron state *s*_*t*_ of the network at this time is expressed by the following equation:

(1) $$\begin{array}{c} s_{t}=\varphi \left(Ux_{t}+Ws_{t-1}\right). \end{array}$$

The network state *s*_*t*_ at time *t* is not only input to the network state at the next time *t*+1 but also the network output at that time. Of course, *s*_*t*_ cannot be output directly, and a coefficient *V* must be multiplied before output, and for the convenience of error back propagation, the output is usually normalized, that is, the output is softmaxed. Therefore, the output *o*_*t*_ equation of the network at time *t* is as follows:

(2) $$\begin{array}{c} o_{t}=\phi \left(Vs_{t}\right). \end{array}$$

Then,

(3) $$\begin{array}{c} \left\{\begin{array}{c} s_{t}^{*}=Ux_{t}+Ws_{t-1}⟶s_{t}=\varphi \left(s_{t}^{*}\right),\\ o_{t}^{*}=Vs_{t}⟶o_{t}=\varphi \left(o_{t}^{*}\right). \end{array}\right. \end{array}$$

The loss function of RNN selects cross entropy, and its calculation equation is as follows:

(4) $$\begin{array}{c} L=-\sum_{i=0}^{n}y_{i}\ln\;y_{i}^{*}, \end{array}$$

where *y*_*i*_ is the true label value and *y*_*i*_^*∗*^ is the predicted value given by the model. Since the RNN model deals with the sequence problem, its model loss can not only be the loss of one moment but also should include the loss of all *N* moments. Therefore, the calculation equation of the loss function of the RNN model at time *t* is as follows:

(5) $$\begin{array}{c} L_{s_{t}}=-\left[y_{t}\ln\left(o_{t}\right)+\left(y_{t}-1\right)\ln\left(1-o_{t}\right)\right]. \end{array}$$

Then, the calculation equation of the global loss for all N moments is as follows:

(6) $$\begin{array}{c} L=\sum_{t=1}^{N}L_{s_{t}}=-\sum_{t=1}^{N}\left[y_{t}\ln\left(o_{t}\right)+\left(y_{t}-1\right)\ln\left(1-o_{t}\right)\right]. \end{array}$$

### 3.4. Self-Attention Mechanism

The attention mechanism is modeled after the internal process of the biological observational behavior, which aligns internal experience with external sensation to increase the fineness of observation in some areas. Because it can quickly extract the important features of sparse data, the attention mechanism is widely used in natural language processing tasks, particularly in machine translation. The self-attention mechanism is an enhancement of the attention mechanism that reduces reliance on external information and improves the ability to capture the internal correlation between numbers and features.

As shown in Figure 3, the essence of the attention function can be described as a mapping from a query to a series of (key value) pairs. In general, a self-attention module has input *n* and output *n*. The self-attention mechanism allows the inputs to interact with each other and find areas where they should pay more attention. The output is the sum of these interactions and attention scores. The calculation equation of self attention is as follows:

(7) $$\begin{array}{c} A\left(Q,K,V\right)=\text{soft }\max\left(\frac{QK^{T}}{\sqrt{d_{k}}}\right)V. \end{array}$$

### 3.5. Proposed Prediction Model

As shown in Figure 4, this paper proposes a smart predictive analysis model for chronic diseases based on self-attention-guided recurrent neural networks and motion perception. The self-attention mechanism layer is added to the RNN in this study, which helps the classification algorithm pay more attention to the internal correlation of its own characteristics. Simultaneously, it collects clinical data and sports data using wearable inertial sensors, which can extract sports data to characterize sluggishness.

## 4. Experiments

### 4.1. Parameter Settings

All algorithm experiments are carried out on a computer with a single NVIDIA GTX1080 GPU (8 GB). The model was built using the TensorFlow deep learning library. Python 3.6.5 is the programming language we use, and 200 samples are processed in batches each time. In addition, the specific parameters are shown in Table 1.

### 4.2. Dataset

The data used in this article comes from Parkinson's Progression Markers Initiative (PPMI) database. PPMI is the first global collaborative project composed of researchers, funders, and research participants, dedicated to identifying biomarkers to improve the treatment of Parkinson's disease. They are committed to establishing standardized protocols for data acquisition and analysis to promote a comprehensive understanding of PD.

### 4.3. Evaluation Index

This article uses precision, accuracy (ACC), F1 value, recall, and AUC (area under curve) as the criteria for evaluating the pros and cons of the classification results. Their calculation equations are as follows:

(8) $$\begin{array}{c} \text{precision}=\frac{\text{TP}}{\text{TP}+\text{FP}},\\ \text{recall}=\frac{\text{TP}}{\text{TP}+\text{FN}},\\ \text{ACC}=\frac{\text{TP}+\text{TN}}{\text{TP}+\text{TN}+\text{FP}+\text{FN}},\\ F1=\frac{2\text{TP}}{2\text{TP}+\text{FP}+\text{FN}}, \end{array}$$

where TP, TN, FP, and FN represent the positive samples with correct judgments, the negative samples with correct judgments, the positive samples with wrong judgments, and the negative samples with wrong judgments, respectively.

### 4.4. Experimental Results

Table 2 shows the PD identification prediction results. It can be seen from the table that the recall rate and F1 value of the proposed algorithm are 71.25% and 83.99%, respectively, which are superior to other algorithms in these indicators. The classification accuracy and specificity of CNN are both 89.23%, which is higher than the other three classifiers. As a result of ACC performance, we reached 93.55%. In this comparison, it is not difficult to find that the ACC of SVM, MPL, LR, and ELM is generally higher than that of CNN, but the F1 value is generally lower than these two deep learning algorithms. This may be caused by an unbalanced relationship in the PD data sample, so ACC cannot be considered unilaterally, and the F1 value should be combined as a measurement standard. Considering the F1 value, ACC, and other values comprehensively, it can be found that the proposed model is better than other methods in overall performance.

### 4.5. Ablation Experiment for Self Attention

In order to further prove the effectiveness of self-attention, we added the ablation experiment of self-attention. “No-self-attention” represents the absence of self-attention mechanism, and “self-attention” represents the use of self-attention mechanism. The ablation experiment results are shown in Table 3.

It can be seen from Table 3 that self-attention is better than no-self-attention in the four evaluation methods. This proves the effectiveness of the self-attention mechanism in the proposed algorithm.

## 5. Conclusion

In this paper, we propose a new type of recurrent neural network classification model based on self-attention mechanism and motion perception to improve the performance of Parkinson's chronic disease recognition and prediction. This model uses a self-attention mechanism and a cyclic neural network to categorize and train the five brain area features retrieved from MRI and DTI images (cerebral gray matter, white matter, cerebrospinal fluid density, and so on). It also uses wearable inertial sensors to gather clinical data, and the motion data can be used to identify characteristic properties that describe slow motion. The findings of the experiments suggest that the self-attention mechanism and the LSTM sequence module successfully improve Parkinson's disease recognition skills.

## Figures and Tables

**Figure 1:** Schematic diagram of the inertial sensor wearing position.

**Figure 2:** Schematic diagram of RNN structure.

**Figure 3:** Schematic diagram of attention mechanism.

**Figure 4:** Schematic diagram of attention mechanism.

**Table 1:** Hyperparameter setting.

Type	Hyperparameter
Adam	lr = 0.0001
	bata_1 = 0.99
	bata_2 = 0.999
	Epsilon = 1e-08
	Decay = 3e-8

**Table 2:** Comparison of prediction results of different algorithms.

Methods	Precision	Recall	F1	ACC
SVM	49.36	52.36	51.23	89.12
MLP	61.21	62.35	69.33	91.25
ELM	45.58	52.36	58.78	90.23
CNN	89.23	69.26	81.25	82.25
Ours	92.36	71.25	83.99	93.55

**Table 3:** Results of self-attention ablation experiments.

Methods	Precision	Recall	F1	ACC
No-self-attention	91.11	70.87	79.58	92.58
Self-attention	92.36	71.25	83.99	93.55

## Data Availability

The data used to support the findings of this study are available from the corresponding author upon request.
